The article "Virtual clinic in pregnancy and postpartum healthcare: A systematic review" was retracted in 2023. Reasons: compromised peer review; unreliable results or conclusions.

# Virtual clinic in pregnancy and postpartum healthcare: A systematic review

**DOI:** 10.1002/hsr2.970

**Published:** 2022-12-21

**Authors:** Ahmadreza Shamsabadi, Mohsen Dashti, Afsaneh Ghasemzadeh, Esmaeil Mehraeen, Ashraf Saber Mashhad Taraqi, Aliakbar Jalali, Zahra Pashaei, Alireza Pashaei

**Affiliations:** ^1^ Department of Health Information Technology Esfarayen Faculty of Medical Science Esfarayen Iran; ^2^ Department of Radiology Tabriz University of Medical Sciences Tabriz Iran; ^3^ Department of Health Information Technology Khalkhal University of Medical Sciences Khalkhal Iran; ^4^ Instructor of Midwifery Education, School of Medical Sciences Esfarayen Faculty of Medical Sciences Esfarayen Iran; ^5^ Faculty of Mechanical Engineering University of Tehran Tehran Iran; ^6^ School of Nursing University of British Columbia Vancouver Canada; ^7^ Iranian Research Center for HIV/AIDS Tehran University of Medical Sciences Tehran Iran; ^8^ Faculty of Electrical and Computer Engineering University of Tabriz Tabriz Iran

**Keywords:** care, postpartum, pregnancy, virtual clinic

## Abstract

**Background and Aims:**

To monitor the health status of pregnant women moment by moment, new technologies in the field of telemedicine can be used, such as virtual visits and virtual clinics. During the COVID‐19 pandemic, by using these technologies, useful and satisfactory services have been provided to pregnant mothers. The aim of this study is to specify the applications, features, and infrastructure of a comprehensive virtual clinic in the field of gynecological and pregnancy care.

**Methods:**

A systematic review search was conducted through the scientific databases from February 2013 to February 2022 using Scopus, Web of Science, and PubMed. Furthermore, manual searches in Google Scholar and the reference lists of included studies were carried out.

**Results:**

In this systematic review we included 16 articles that reported experiences in virtual clinics in pregnancy and postpartum healthcare. The involved studies were experimental, cohort, and cross‐sectional studies. The target group users were pregnant or women who gave birth and families of neonatal. The application of virtual clinics was for the visit, consultation, monitoring, follow‐up, and home care virtually. Highly satisfaction scores of caregivers after virtual visits and consultation were reported. There were some challenges during virtual visits and consultation; the most important challenge was a poor internet connection.

**Conclusion:**

The reviewed studies show promising outcomes according to patient and provider satisfaction. We predict that telehealth will become a growingly significant part of gynecological care in the future.

## 1 INTRODUCTION

Prenatal care and infant mortality rates have been identified as one of the quality indicators of care provision by the World Health Organization, while more than 44 million women in developing countries still do not have access to such cares.^1^ Factors such as pregnancies in old ages (high‐risk pregnancies) and unmanaged diet increase the risk of developing hypertension and diabetes during pregnancy.^2^ On the other hand, due to the presence of chronic diseases in pregnant women, the need for continuous monitoring of the health status of them during pregnancy is inevitable.^3^, ^4^ To screen the health situation of pregnant women moment by moment, new technologies in the field of telemedicine can be used, such as virtual visits and virtual clinics.^5^, ^6^ Virtual clinics have benefits such as continuous monitoring of vital and clinical signs, saving time in providing care, reducing hospitalization and paraclinical costs, and increasing patient satisfaction.^7^ Although telemedicine has grown in recent years, particularly to provide access to specialized care for patients living in rural or remote communities, telemedicine has rarely been utilized in prenatal care.^8^ Also, before the COVID‐19 pandemic, telemedicine was not routinely used in obstetrics. However, after the declaration of a state of emergency due to COVID‐19, the American College of Obstetricians and Gynecologists (ACOG) advised to arrange some appointments in the style of “telehealth” to decrease transmission of infection during clinic visits or due to having a meeting with healthcare staff.^9^ During the COVID‐19 pandemic, by using these technologies, useful and satisfactory services have been provided to pregnant mothers through virtual visits and health monitoring.^10^, ^11^ According to the searches conducted in the databases, scattered studies have been conducted on the use of virtual clinics for prenatal care focusing on the applications, capabilities, and infrastructure of virtual clinics for pregnant women. The purpose of this study is to specify the applications, features, and infrastructure of a comprehensive virtual clinic in the field of gynecological and pregnancy care.

## 2 METHODS

This systematic review was carried out compliant with to the Preferred Reporting Items for Systematic Reviews and Meta‐Analyses (PRISMA) guidelines.^12^ Systematic searches were done in the scientific online databases using selected keywords from February 2013 to 2022.

### 2.1 Data sources

We performed a systematic search using three databases including Scopus, Web of Science, and PubMed. Also, we conducted manual searches in the reference lists and Google Scholar.

### 2.2 Search strategy

Search strategies were written by the first and corresponding authors. Search terms are performed in a highly‐delicate method via the Boolean operator OR. The search strategy is defined as follows:

A. Pregnancy OR gestation OR prenatal OR perinatal OR neonatal OR antenatal OR childbirth OR “delivery care” OR postnatal OR postpartum OR “midwifery care” OR “maternal health” OR “postpartum program.”
B. Telemedicine OR telehealth OR telecare OR telemonitoring OR telehomecare OR teleconsultation OR tele‐education OR “m‐health” OR “e‐health OR” “virtual visit” OR “virtual clinic” OR “virtual care” OR “virtual health.”
C. [A] AND [B].

### 2.3 Eligibility criteria

The original and English studies that reported the design and implementation of the virtual clinic and virtual visit in maternal care were included. We considered the following exclusion criteria:

(1) Non‐original studies, including conference abstracts, review articles, protocols, and editorial.
(2) Ongoing clinical trials.
(3) Unavailability of full texts.
(4) Original articles that don't report the design, implementation, and application of virtual clinic in maternal care.

### 2.4 Selection study and data screening

We used the EndNote software version 9.0 to manage the retrieved studies. A single EndNote library was used to combine search results and duplicate studies were deleted. The articles were screened independently by two authors of the research team in different steps. First, the title and abstract of the studies were screened and the ineligible articles were deleted. Then, they investigated the full text of the remaining articles based on inclusion and exclusion criteria and the eligible articles were recognized.

### 2.5 Data extraction

Required data were extracted by three authors of the research team as follow: first author, type of study, country target group users, applications, capabilities, infrastructures, benefits, challenges summary of findings. They managed the results of included articles in Table 1. The first author investigated the extracted data and settled any disagreements among the other authors.

**Table 1:** Applications, benefits, and challenges of the virtual clinic in prenatal healthcare

ID	First author (reference)	Type of study	Country/year	Target group users	Purpose of virtual clinic	Capabilities	Infrastructures	Benefits	Challenges
1	HaikalSatria^28^	Experimental	Malaysia 2014	Pregnant women	Virtual prenatal visit	Two‐way communication	Wireless Mesh Network, Medical Data Assistant (MDA), Medical Device Interface (MDI), microphone, camera, ECG, Doppler instrument, blood pressure monitor, ultrasonic machine, and stethoscope	low‐cost application in emergency time, acceptable medical data transfer quality	Maximum 1 km transmission distance
2	Garne et al.^13^	Experimental	Denmark 2016	Family of neonatal with tube feeding	Identify parental needs and provide home care with telemedicine	N/A	Video conferencing	Giving parents the feeling of being family, promote self‐efficacy of parents, receive guidance when they need, a positive effect on parent‐infant relationship, feeling of security for parents because of having initiative for infant care	N/A
3	Pflugeisen et al.^14^	Experimental	USA 2016	Low‐risk pregnant women	A combine of in‐person and virtual visits in prenatal care with OB Care Connect™	Six prenatal visits, blood pressure, the body weight of mother, rate, rhythm, and regularity of the fetal heart tones with obstetric advanced registered nurse practitioner	Video conference	N/A	N/A
4	Deldar et al.^15^	Experimental	Iran 2017	High‐risk pregnant women	Tele‐decision‐making clinical archetypes for management of high‐risk pregnancies	N/A	Telephone	Better data quality, adequacy, organization, confidence, and convenience	Lack of specific structure
5	Rhoads et al.^16^	Experimental	USA 2017	Preeclampsia pregnant women	m‐health	Monitor blood pressure, weight, pulse, and oxygen saturation	m‐health device (Ideal Life equipment), Bluetooth, wireless, cloud‐based caregiver portal	Returned to healthcare facilities if needed, safely manage during the postpartum period	N/A
6	Pflugeisen et al.^17^	Experimental	USA 2017	Pregnant women	Virtual visit with video conference	Blood pressure	Doppler monitor, blood pressure cuff	Highly satisfied with the care	N/A
7	Alves et al.^18^	Experimental	Brazil 2019	High‐risk pregnant women	Tele‐monitoring	Blood pressure, sign, and symptoms, accompanying charts, alerts	A prototype of gestational hypertensive syndromes module	Low cost, high impact intervention, continuous monitoring, early intercurrent screening, better screening for high‐risk pregnant women	N/A
8	Wichman et al.^19^	Experimental	USA 2019	Pregnant women	Psychiatric teleconsultation	N/A	Telephone, triage coordinator, text messaging, email, pager	All of the respondents were strongly satisfied with the services	Availability of psychiatric
9	Krenitsky et al.^10^	Experimental	USA 2020	COVID‐19 infected pregnant women	Virtual visit with video conference	Temperature, heart rate, oxygen saturation, blood pressure, qualitative fetal movement assessment, and fetal kick counts	Thermometers, blood pressure cuffs, portable pulse oximeters, telephone, smart devices	N/A	Inconsistent follow‐up, poor connection
10	Curfman et al.^20^	Cohort	USA 2020	Pediatric transport team	Telemedicine for a consult for transferring children to a hospital	Patient's symptoms and sign	Mobile device (video or phone communication), Wi‐Fi, a cellular connection	Changed patients outcome or management	Connectivity
11	Bishop et al.^21^	Experimental	USA 2020	Patients with fetal anomalies	Telehealth visit and follow‐up	N/A	HIPPA‐secure platform, video visit, telephone	Decrease time and expenses burden, increased access to patient	Poor connection, lack of internet access, lack of proper smart device
12	Jakubowski et al.^22^	Cross‐sectional	Poland 2021	Pregnant or gave birth to women, age group of 18−40	Virtual visit and follow‐up	N/A	Social media, the internet	Better and more complete follow‐up during pregnancy	N/A
13	Campbell‐Yeo et al.^23^	Experimental	Canada 2021	Families of neonatal	Optimal care for NICU families	Provide education through virtual evidence‐based resources	Video conferencing system	Standardized, equitable, and transparent care to increase parent engagement	Feeling overwhelmed by family in the initial days, increased workload of nurses
14	Reisinger‐Kindle et al.^24^	Cohort	USA 2021	Pregnant women	Telehealth visit	Two‐way communication	Video conferencing, telephone	Satisfaction of caregivers	Less screening documents
15	Nelson et al.^25^	Cohort	USA 2021	Pregnant women	Telehealth visits for routine care	Weight, blood pressure, fetal heart tone	Doppler monitor	Satisfaction of caregivers, improved self‐care abilities	The cost associated with renting or purchasing equipment
16	Palmer et al.^26^	Experimental	Australia 2021	Pregnant women	Telehealth service and consultation	Endocrinology consultations, blood pressure, blood glucose	Smart devices, telephone	Low cost	N/A

Abbreviation: OGTT, oral glucose tolerance test.

### 2.6 Quality assessment

This systematic review study used the PRISMA guideline to evaluate articles. The quality of the studies was surveyed by three independent and experienced authors. Any discrepancies in the quality of the selected studies between authors were judged by the first author and agreed with the majority. To assess the quality of the included studies the Newcastle−Ottawa scale was used (Table 2).^27^ According to three categories of selection, comparability, and outcome a maximum number of 9 was assigned to studies.

**Table 2:** Newcastle−Ottawa scale quality assessment of the study

First author	Selection (out of 4)	Comparability (out of 2)	Exposure/outcome (out of 3)	Total (out of 9)
Dominik Jakubowski^22^	***	**	**	7
Muhammad Haikal Satria^28^	***	*	***	7
Marsha Campbell‐Yeo^23^	****	**	***	9
Kolsoum Deldar^15^	****	**	***	9
Keith Reisinger‐Kindle^24^	***	**	***	8
Sarah J. Rhoads^16^	***	*	***	7
Christina L. Wichman^19^	**	**	**	6
Gretchen A. Nelson^25^	****	**	***	9
Alison Curfman^20^	***	**	***	8
Bethann Mangel Pflugeisen^17^	***	**	***	8
Christine E. Bishop^21^	****	**	**	8
Nicole M. Krenitsky^10^	***	**	***	8
Danielle Santos Alves^18^	***	**	***	8
Kristina Garne^13^	****	**	**	8
Bethann M. Pflugeisen^14^	***	*	***	7
Kirsten R. Palmer^26^	***	**	***	8

*Note*: *, **, ***, **** means score 1, 2, 3, and 4 respectively.

## 3 RESULTS

We reviewed the available evidence on the virtual clinics in pregnancy and postpartum healthcare. For this purpose, 55 articles were identified. Out of them, 24 articles were removed because of duplication and 31 articles were screened. Based on the inclusion and exclusion criteria, 7 article was deleted and finally, the full text of 16 articles were reviewed. The selection process of articles is shown in the PRISMA diagram (Figure 1). Most of the studies have been done in the United States of America (*n* = 9) and one study in each of the countries of Iran, Poland, Malaysia, Canada, Brazil, Denmark, and Australia. The involved studies were as follow: experimental (*n* = 12), cohort (*n* = 3), and cross‐sectional (*n* = 1) studies.

**Figure 1:** Search results from different databases

The target group users were pregnant or women who gave birth and families of neonatal. The application of virtual clinics was for the visit, consultation, monitoring, follow‐up, and home care virtually. The virtual clinics provide two‐way communication between patient and caregivers, education via virtual resources, tele‐monitoring sign and symptoms of pregnant women (including oxygen saturation, pulse rate, blood pressure, blood glucose, and weight), and fetal movement assessment. Also, in the combined methods of in‐person and virtual visits, fetal heart tone and ultrasound of pregnant women were assessed. The infrastructure required for the virtual clinic has been reported as follows: smart devices, telephone, pager, microphone, camera, internet (Wi‐Fi, cellular connection), Wireless Mesh Network, medical data assistant, and medical equipment (Doppler monitor, portable pulse oximeters, blood pressure cuffs, thermometers).

Studies have reported numerous benefits from virtual clinic experiences; in a cross‐sectional study conducted among 18−40 years old pregnant or gave birth women, Jakubowski et al.^22^ mentioned better and more complete follow‐up as benefits of virtual visits during pregnancy. Some studies reported high satisfaction scores of caregivers after virtual visits and consultation.^17^, ^19^, ^24^, ^25^ Two studies reported that during the virtual visit, patients who needed more treatment and care were immediately referred to medical centers and possible complications for the mother and fetal/neonatal were avoided.^16^, ^20^ Other advantages were low cost,^18^, ^21^, ^26^, ^28^ standardized, equitable, and transparent care,^23^ better screening for high‐risk pregnant women,^18^ better data quality,^15^, ^28^ and giving parents the feeling of being family.^29^ There were some challenges during virtual visits and consultation; the most important challenge was poor internet connection,^10^, ^20^, ^21^ following lack of specific structure for implementation of virtual clinics,^15^ lack of screening documents due to personnel inconsistency, and forgetting to record information,^24^ lack of availability of specialist doctors and psychiatrists,^19^ and high cost of renting or purchasing medical equipment for tele‐monitoring.^25^

## 4 DISCUSSION

This review was conducted due to the growing use of telemedicine in prenatal, neonatal, and postpartum care. We included studies that established virtual systems, either hybrid care or substitute for in‐person care. Overall, no significant difference was seen between in‐person and virtual care in terms of satisfaction, patient, and provider outcome. Virtual care has been showed promising results for managing and monitoring high‐risk pregnancies. After the declaration of a state of emergency due to COVID‐19, to decrease transmission of infection holding visit meetings in the form of “telehealth” was recommended by ACOG,^9^ thus the number of appointments has been reduced which on one hand, resulted in saving time, costs, and higher patients and providers satisfaction but on the other hand faced new challenges and required infrastructures. We will further discuss our findings in‐depth.

### 4.1 Appointments

Telemedicine interventions may reduce appointments for in‐person prenatal care visits. The latest ACOG guidelines^9^ suggested about 12−14 gynecological care visits, but several studies investigated a reduction from 14 patient visits according to 9 or even fewer visits because of the use of virtual nurse‐midwife and physician visits, and remote monitoring for women with low‐risk pregnancies.^14^, ^17^, ^22^, ^24^, ^25^, ^26^ Different virtual visit schedules were developed by studies but the main frame was the same; after initial evaluation for enrollment by a physician, particular pregnancy milestones (i.e., the 8‐ and 20‐week ultrasound, prenatal labs) were in‐person visits and also the number of in‐person visits increased with gestational age, due to the higher possibility of incidence of pregnancy complications.^17^ Similar missed appointments numbers were detected for both in‐person and virtual appointments. However, the influencing factors may be different. In‐person visits may be affected by concerns about exposure to COVID‐19 and the challenges of attending during quarantine, while challenges related to technology, communication, and accessibility issues may affect attending virtual visits.

### 4.2 Infrastructures

To perform virtual visits, basic equipment items and infrastructures are essential. Healthcare providers (HCPs) require a computer or laptop, tablet, or smartphone with video call capabilities with internet service. Patients can use a smartphone, tablet, or computer with the same capabilities to carry out remote monitoring, remote image transmission, education, triage, consultation, and interpretation of ultrasounds and non‐stress tests. Mobile phone applications are mostly used for remote monitoring and education.^16^ Additionally, specific portable items are needed during virtual visits like blood pressure cuff, portable pulse oximeter, home Doppler, tape measure, glucometers, and mobile cardiotocograph devices. With the help of providers, pregnant women can check fundal heights, serial blood pressures and weights, fetal kick counts, fetal heart rate, and uterine contractions. The telehealth appointments required pregnant women to learn how to use these devices.^25^ However, Doppler tones and also, non‐stress tests for fetal monitoring couldn't be acquired for home use owing to the lack of reliable and commercially available remote monitoring equipment, but the qualitative assessment of fetal movement and the number of fetal kicks were possible to evaluate fetal well‐being.^10^ The data derived from these devices and a series of symptom‐related questions were recorded on an electronic medical record platform or a cloud‐based database by HCPs.^10^ The costs of these equipment and funding resources haven't been mentioned in the studies; they may be purchased by patients, rented by hospitals, or provided by funding resources.

### 4.3 Consultation

Besides reducing the number of in‐person visits, assessment of fetal well‐being, and monitoring and limiting weight gain, that is, consultation is one of the common benefits and usages of telemedicine which has been used for several years in prenatal care. Teleconsultation can be easily performed with subspecialties such as cardiology, anesthesiology, psychology, and endocrinology.^15^, ^21^, ^26^ Wichman et al.^19^ performed 504 psychiatric teleconsultations for diagnosis, treatment, and management of perinatal women who have any psychiatric disorder or history of substance abuse which lead to 100% provider satisfaction with the service. Palmer et al. found their telehealth program provided about half of antenatal consultations via telehealth and did not affected the detection and management of common complications of pregnancy, including fetal growth restriction, preeclampsia, and gestational diabetes.

### 4.4 High‐risk

Expanding principles of telemedicine is not only used for routine prenatal care but also for management of high‐risk pregnancies. Hypertensive disorders of pregnancy are one of the leading factors of maternal mortality worldwide by affecting 2% to 8% of pregnancies in both developing and developed countries.^30^, ^31^ One of the main purposes and important aspects of virtual visits which most of the included studies in this paper performed was checking and monitoring blood pressure with a home cuff that is effortlessly available at local pharmacy stores or online.^10^, ^14^, ^16^, ^17^, ^18^, ^25^, ^26^, ^28^ High‐risk pregnancies with hypertension‐related disorders such as gestational hypertension, preeclampsia, chronic hypertension, and eclampsia have also been remotely managed and monitored in prenatal and postpartum periods by virtual visits.^15^, ^18^ Rhoads et al.^16^ used mobile health (m‐health) technologies to closely manage 50 women diagnosed with preeclampsia during the postpartum period. There was no statistical difference in satisfaction, benefits, and ease of use in comparison to the control group. In the virtual visit program of Pflugeisen et al., 5 of the 15 visits (14 prenatal and 1 postpartum in Week 42) were performed via video conference with an obstetric advanced registered nurse practitioner. Virtual visit patients had higher incidence of preeclampsia was higher (8.5% vs. 3.4%). Thus, the researchers did not comment on potential reasons for the increased rate of preeclampsia in virtual visit patients.^14^

### 4.5 Challenges

Barriers to telehealth are fall into two main categories: the first and most important which is largely mentioned in the included studies is providing a safe, dependable connection between providers and patients. Poor connection causes loss of communication and frustrated patients and providers. Pflugeisen et al.^14^ mentioned ease and quality of connection as a key role in overall patient satisfaction. The main reasons were as follow: the provider or patient technical problems, poor or lack of internet access, and lack of proper smart device.^10^, ^20^, ^21^ A significant start‐up cost is another barrier that is necessary to perform telehealth, which can be the main barrier to begin with.^32^ Some other barriers include lack of knowledge about technology, lack of trust, conservative attitude, and the belief that telehealth visits are unsentimental.^32^ Krenitsky et al.^10^ explained technological difficulties of using video technology by patients as a significant barrier. Also, Doppler tones and non‐stress tests for fetal movement evaluation couldn't be assessed due to a lack of reliable and commercially available equipment.^33^ Curfman et al.^20^ interpreted barriers by division; they showed a poor internet connection, desktop station difficulty, mobile app difficulty, and environmental background noise in divisions of Children's Direct, emergency department, NICU, PICU, and transport team. The mean perceived usefulness, hindrance, and by division, burden of telemedicine varied significantly.

### 4.6 Effects of COVID‐19 on telehealth

The COVID‐19 pandemic has been a fuel for change in prenatal care delivery by reducing traditional in‐person visits at the first step, and also by increasing funding for telehealth services. The in‐person visits limitations are due to parental presence restrictions and constantly‐changing COVID‐19 policies guidelines, which lead to missed appointments.^34^, ^35^ An properly performed telehealth system can guarantee that pregnant patients with COVID‐19 receive sufficient visits and monitoring which can be equal to in‐person care. Telehealth allows patients with mild COVID‐19 to stay physically out of health settings and protect other patients and HCPs from exposure to COVID‐19 patients.^10^

### 4.7 Virtual‐ versus in‐person visits outcomes

There is an apparent concern that a decrease in traditional in‐person visits may cause lower satisfaction of patients and lower quality of care. In 2017, Pflugeisen et al.^17^ conducted a randomized trial of 430 virtual visits, in which some of parental care of patients delivered via virtual visit. Patients declared significantly higher rate of satisfaction by this hybrid model of care compared with traditional care. Reisinger‐Kindle et al.^24^ did not use formal surveys and interviews to assess provider satisfaction with telehealth due to the crisis during the COVID‐19 pandemic. However, Wichman et al.^19^ showed 100% provider satisfaction with the perinatal psychiatric teleconsultation via self‐reported online surveys. In a study in 2019 by Butler Tobah et al.,^36^ in a randomized study, reduced prenatal visit model with virtual visits or usual care in women was assessed. The reduced hybrid model consist of 8 in‐person and 6 virtual visits. Results showed that the reduced hybrid model saved 2.8 prenatal visit per patient. The women in the virtual care group had significantly higher satisfaction, lower pregnancy‐related stress, and even lower healthcare costs.

### 4.8 Experience

The majority of the women who intended the virtual care were recommending it to others. However, Pflugeisen et al.^17^ found that women who were in their first pregnancy may be significantly less likely to participate in virtual visits than women who are already mothers. Nelson et al.^25^ showed that the virtual visit experience was comparable and admissible to the traditional in‐person appointments for both patients and providers. Wichman et al.^19^ reported 100% provider satisfaction with teleconsultation.

### 4.9 Safety

Telehealth demonstrated to be an efficient option concerning patient safety. Several studies did not report significant differences in complications including, preterm delivery, cesarean deliveries, or birthweight among patients who received traditional prenatal care and those who received telehealth visits.^14^, ^17^ A significantly higher rate of preeclampsia in patients receiving virtual visits reported by one study (8.5% vs 3.4%). However, no significant difference between traditional and virtual visits in other outcomes including gestational diabetes mellitus, mean birthweight, preterm birth, NICU admissions, gestational age at birth, and cesareans were reported.^14^

## 5 LIMITATION

This review has several important limitations. Most of the studies were done in the United States which reflects the socioeconomical need to implement telehealth worldwide. The majority of included women in the studies were white women who were generally educated and had higher socioeconomic status (SES). As expected, most of the studies had a low sample size, unequal sizes of the comparison groups, and only included low‐risk pregnancies. Further studies should include a larger population with different ethnicities and SES to evaluate maternal and neonatal adverse events and maternal mortalities compared to the standard care group.

A major limitation of included studies was their lack of data on provider productivity and reduction of costs. None of the studies reported the cost effectiveness of virtual visits. There was no information about funding resources, or purchasing or renting equipment. As their first experience, the main goals of these studies were mainly to assess the safety, and satisfaction of the implementation of virtual visits for mothers and babies.

## 6 LOOKING FORWARD

Results of the present study showed that virtual health is changing the healthcare landscape, and to stay competitive and on‐use by patients, the traditional healthcare business models will need to be evolved. It is recommended to carry out further studies to investigate the impact of the virtual clinic on the total costs of treatment and the overall costs of establishing virtual clinics to show whether or not virtual clinics are economical in general.

## 7 CONCLUSION

This review emphasizes the increasing use of telemedicine in obstetrics. It specifically evaluates telehealth infrastructures and types of interventions that improve existing prenatal care systems. The reviewed studies show promising outcomes according to patient and provider satisfaction. We predict that telehealth will become a growingly important part of obstetric care in the future. However, barriers such as technology and maintaining quality will continue to require attention highlighting the importance of reliable support and infrastructure.

## AUTHOR CONTRIBUTIONS

**Ahmadreza Shamsabadi**: Conceptualization; project administration; supervision; writing – original draft. **Mohsen Dashti**: Data curation; investigation; methodology; writing – original draft. **Afsaneh Ghasemzadeh**: Data curation; investigation; methodology; validation; writing – original draft. **Esmaeil Mehraeen**: Data curation; investigation; validation; writing – review & editing. **Ashraf Saber Mashhad Taraqi**: Methodology; writing – original draft. **Aliakbar Jalali**: Data curation; methodology; writing – original draft; writing – review & editing. **Zahra Pashaei**: Conceptualization; investigation; project administration; supervision; writing – original draft; writing – review & editing. **Alireza Pashaei**: Investigation; methodology; project administration; writing – original draft; writing – review & editing. All authors have read and approved the final version of the manuscript

## CONFLICT OF INTEREST

The authors declare no conflict of interest.

## ETHICS STATEMENT

The Ethics Committee of Esfarayen University of Medical Sciences approved the study (Approval No. IR.ESFARAYENUMS.REC.1399.037).

## TRANSPARENCY STATEMENT

The lead author Zahra Pashaei, Alireza Pashaei affirms that this manuscript is an honest, accurate, and transparent account of the study being reported; that no important aspects of the study have been omitted; and that any discrepancies from the study as planned (and, if relevant, registered) have been explained.

## Data Availability

The authors stated that all data underlying the results presented are available in the article. Alireza Pashaei and Zahra Pashaei had full access to all of the data in this study and take complete responsibility for the integrity of the data and the accuracy of the data analysis.
